# The Application Value of ceMDCT in the Diagnosis of Gastric Cancer Extramural Vascular Invasion and Its Influencing Factors

**DOI:** 10.1155/2022/4239600

**Published:** 2022-01-07

**Authors:** Shifeng Yang, Xiaoming Zou, Jiacheng Li, Ange Zhang, Lei Zhu, Xiaolong Hu, Changjian Li

**Affiliations:** Department of Gastrointestinal Surgery, The Second Hospital of Harbin Medical University, Harbin, China

## Abstract

**Objective:**

To investigate the value of enhanced multislice spiral CT (ceMDCT) in the diagnosis of extramural vascular invasion of gastric cancer and the influencing factors of extramural vascular invasion. There are different methods used in this paper.

**Method:**

131 patients with primary gastric cancer treated in our hospital from January 2017 to May 2019 were selected. All patients underwent surgical resection and ceMDCT examination before operation.

**Result:**

There were 40 cases with extramural vascular invasion of gastric cancer by surgical pathological diagnosis. The kappa value of ceMDCT in diagnosing extramural vascular invasion of gastric cancer was 0.947, and the consistency was excellent. The diagnostic sensitivity, specificity, positive predictive value, and negative predictive value were 100.00%, 96.70%, 93.02%, and 100.00%, respectively. The proportions of T3-T4, tumour diameter ≥5.0 cm, and growth pattern of proximal nodular + diffuse type in patients with gastric cancer extramural vascular invasion were 92.50%, 85.00%, and 65.00%, respectively, which were significantly higher than those in patients without extramural vascular invasion (*P* < 0.05). The logistic regression analysis results showed that T3-T4, tumour diameter ≥5.0 cm, proximal nodular + diffuse growth pattern were the risk factors for extrahepatic vascular invasion in gastric cancer (OR = 3.751, 2.901, and 3.367, *P* < 0.05).

**Conclusion:**

ceMDCT has good application value in diagnosing gastric cancer extramural vascular invasion. The occurrence of gastric cancer extramural vascular invasion is affected by T staging, tumour diameter, and tumour growth pattern.

## 1. Introduction

Gastric cancer is a malignant tumour originating from the epithelium of the gastric mucosa and is the most common of all malignant tumours of the digestive tract [1]. Gastric cancer has the characteristics of unobvious early symptoms and poor prognosis. Patients are already in the middle and late stages of gastric cancer when they are diagnosed, and the treatment is difficult. The most common clinical treatment is surgical resection of the lesion [2]. Extramural vascular invasion is a common complication of gastric cancer, which refers to the distant spread of the tumour into veins outside the gastrointestinal muscular layer, with an incidence rate of about 30% [3]. It is important to judge whether the patient has extramural vascular invasion before surgery. Because of the different experiences of doctors, the judgment of extravascular invasion is not the same, and the judgment error is also significant. It is not appropriate to use pathology to judge the occurrence of extravascular invasion. Contrast-enhanced multislice spiral CT (ceMDCT) can provide high-resolution images and multiplanar reconstruction techniques. Preoperative imaging technology can diagnose the vascular wall invasion of gastric cancer. Clinically, a comprehensive analysis of ceMDCT imaging and pathology is needed to improve the diagnostic efficacy of the two. This study selected 131 patients with primary gastric cancer treated in our hospital from January 2017 to May 2019 to explore the application value of ceMDCT in the diagnosis of extramural vascular invasion of gastric cancer and its influencing factors.

## 2. Data and Methods

### 2.1. General Information

131 patients with primary gastric cancer treated in our hospital from January 2017 to May 2019 were selected, including 73 males and 58 females; age 21–70 years, median age (51.03 ± 7.22) years; and pathological type: 61 cases of squamous cell carcinoma, 39 cases of adenosquamous carcinoma, and 31 cases of papillary adenocarcinoma. Inclusion criteria: (1) pathologically confirmed; (2) ceMDCT examination and surgical treatment in our hospital; (3) TNM staging refers to the standards in the 8th edition of the TNM staging system for gastric cancer issued by UICC and AJCC [4]; and (4) complete preservation of clinical data. Exclusion criteria: (1) with other malignant tumours; (2) poor image quality; and (3) preoperative radiotherapy and chemotherapy treatment history.

### 2.2. ceMDCT Inspection

Scanning and reconstruction parameters: fasting 8 h before the examination, drinking 600∼800 ml 5 min before the examination, and moderate filling of the gastric cavity. 64-row MDCT (GE USA) was used. MDCT scan parameters were 120 kV, 240–260 mAs, collimation 64–0.6, and slice thickness 5 mm, ranging from the diaphragm to pubic symphysis. After a plain scan, the high-pressure syringe (Ulrich GmbH & Co, Germany) was used for the injection of 100 ml iodine contrast agent (iopromide, German Bayer Xianling Pharmaceutical Company) through the median cubital vein at the injection rate of 2.5 ml/s, the action phase, and portal vein scan. The original image of the portal phase was reconstructed at transverse, sagittal, and coronal positions using the Advantage Workstation 4.3 (GE, USA). The thickness of the reconstructed image layer was 1.25 mm.

### 2.3. Pathological Examination

During the operation, the doctor observed whether the tumour spread with the naked eye, judged the invasion of extravascular blood vessels, and compared it with the preoperative judgment for statistical calculation.

### 2.4. Statistical Treatment

IBM SPSS Statistics 22.0 (SPSS Inc., Chicago, IL, USA) was used for statistical analysis. The experimental data were presented as ACCEPTED MANUSCRIPT mean ± standard deviation (mean ± SD), and the *t*-test was used for count data. The *χ*2 test and kappa test were used with kappa value > 0.75 and excellent consistency; multivariate analysis used logistic regression analysis. One-way analysis of variance was used for comparison of parametric data among groups, followed by Turkey's test for comparison between two groups, while the Mann–Whitney *U* test was performed for difference analysis of nonparametric data, and *P* < 0.05 indicates that the difference is statistically significant.

## 3. Results

### 3.1. Surgical Pathologic Results

After surgical pathological diagnosis, out of 131 patients with gastric cancer, 40 had an external vascular invasion of gastric cancer.

### 3.2. ceMDCT Diagnostic Results

The consistent kappa value of c eMDCT diagnostic extrawall vascular invasion and surgical pathology outcome of gastric cancer was 0.947, with its diagnostic sensitivity, specificity, and positive and negative predicted values of 100.00% (40/40), 96.70% (88/91), 93.02% (40/43), and 100.00% (88/88), respectively, as shown in Table 1, *P*=0.01.

### 3.3. Comparison of Clinical Data of Patients with or without Extramural Vascular Invasion of Gastric Cancer

The group's example number, gender, age, and T, N, and M installment are all shown in Tables 2. We can inform that T3∼T4 tumours with gastric cancer had a significantly higher proximal nodular type + proportion than those with nonvalvular vascular invasion (*P* < 0.05).

### 3.4. Multifactor Analysis

Logistic regression analysis of T stage, tumour diameter, and growth mode as the independent variables and whether gastric cancer wall vascular invasion occurred as the dependent variable showed that T3∼T4, tumour diameter ≥5.0 cm, and proximal nodular + diffuse growth mode were risk factors for extrawall vascular invasion in gastric cancer (**OR** = 3.751, 2.901, and 3.367, *P* < 0.05), as shown in Table 3.

## 4. Discussion

Gastric cancer is a common malignant tumour occurring in the digestive tract. It has the characteristics of minor early clinical symptoms and poor patient prognosis. The survival rate of patients with early gastric cancer is very high. Studies have shown that the survival rate of early gastric cancer is more than 90%, and the survival rate of advanced gastric cancer is far lower than that of patients with early gastric cancer [5]. The incidence of vascular invasion outside the wall of the common complications of gastric cancer is about 30%. Still, because the patient's clinical performance is not obvious, the condition is not easy to diagnose, resulting in the patient's condition gradually aggravating due to the delay and even reducing the patient survival rate [6, 7]. Currently, the standard diagnosis methods in China are still pathologically diagnosed by experienced doctors [8]. However, due to different experiences, sometimes, the misdiagnosis rate is high, affecting patient prognosis and reducing survival rate [9].

It has been shown that extrawall vascular invasion usually coexists with extraspinal nerve and lymphatic vessel infiltration and is a way of tumour spreading along the neurovascular tract [10]. Due to extrawall vascular invasion, tumour cells can spread throughout the portal system and eventually form distant metastasis [11]. The rate of distant metastasis in gastric cancer is positively associated with the degree of venous invasion, and external vascular invasion is an independent risk factor for predicting whether distant metastases occur and the chance of postoperative tumour recurrence [12–14]. Clinically, gene sequencing technology can classify gastric cancer into proximal nondiffuse type, distal nondiffuse type, and diffuse type, and distal nondiffuse type prognosis is significantly better than proximal nondiffuse type and diffuse gastric cancer [15]. The occurrence of extrawall vascular invasion in gastric cancer is closely related to the poor prognosis in gastric cancer patients. It is an independent risk factor for predicting distant metastasis and recurrence [16]. Surgical pathological diagnosis is an effective method to find extrawall vascular invasion, which can detect positive extravascular infiltration, but the results are susceptible to multiple factors and have specific false-negative effects [17].

This study creatively uses medical techniques and CT imaging techniques to diagnose extravascular invasion, and using CT imaging diagnosis can significantly improve diagnostic accuracy [18]; the diagnosis can be seen, and the images can be used to analyze the lesions as well as more intuitively display the diffusion situation, and the stability is improved [19], which is also the innovation of this study. After surgical pathological diagnosis, 40 patients showed external vascular invasion of gastric cancer [20].

In this study, T stage, tumour diameter, and growth mode were taken as independent variables, and whether extravascular invasion occurred was taken as the dependent variable for logistic regression analysis. The results showed that T3∼T4, tumour diameter ≥5.0 cm, and proximal nodular + diffuse growth mode were risk factors for extravascular invasion in gastric cancer. The diagnosis of ceMDCT for external vascular invasion in gastric cancer was associated with T stage, tumour growth mode, tumour size, and pathological stage.

The ceMDCT diagnosis of gastric cancer nonwalled vascular invasion and surgical pathological results were excellent. Its diagnostic sensitivity, specificity, positive predictive value, and negative predictive values were at high levels, and T3∼T4, patients with gastric cancer tumour diameter ≥5.0 cm, and proximal nodular + diffuse growth mode were significantly higher than in patients with nonmural vascular invasion. The analysis is that extravascular invasion of the tumour is based on the spread of the tumour along the nerve vessels. Thus, the larger the tumour, the greater the likelihood of proximal nodular and dispersal vascular invasion. It is shown that abdominal CT examination can be used to determine vascular invasion outside gastric cancer, which can more accurately visualize the patient's lesion and spread by image analysis and accurately observe the extent of tumor invasion and distant organs and lymph node metastases, helping to obtain a clearer diagnostic result.

This study is limited to retrospective imaging characterization, and prospective studies are needed to further determine the relevance of extramural vascular invasion with patient prognosis. The diagnosis of extrawall vessel invasion by preoperative ceMDCT would be an effective indicator of preoperative gastric cancer risk stratification after the TNM stage.

## 5. Conclusions

In conclusion, ceMDCT has good application value in the diagnosis of vascular invasion outside the gastric cancer wall, where vascular invasion is affected by T stage, tumour diameter, and tumour growth mode, and prospective studies are needed to further determine the relevance of extramural vascular invasion with patient prognosis.

## Figures and Tables

**Table 1:** Comparison of ceMDCT and surgical pathological results.

ceMDCT diagnosis	Surgical pathology		Kappa	*P*
	There is extrawall vascular invasion	There is no extracellular vascular invasion		
There is extrawall vascular invasion	40	3	0.947	0.01^*∗*^
There is no extracellular vascular invasion	0	88		

*P* < 0.05 indicates that the difference is statistically significant.

**Table 2:** Comparison of clinical data of gastric cancer.

Group	Example number	Male/female	Age (years)	T installment		N installment		M installment		
				T1∼T2	T3∼T4	N0	N1∼N2	M0	M1	
There is extrawall vascular invasion	40	24/16	50.87 ± 8.03	3 (7.50)	37 (92.50)	11 (27.50)	29 (72.50)	27 (67.50)	13 (32.50)	
There is no extravascular invasion	91	49/42	52.10 ± 9.44	33 (36.26)	58 (63.74)	31 (34.07)	60 (65.93)	66 (72.53)	25 (27.47)	
*t/χ* ^2^		0.426	−0.717	11.536		0.550		0.341		
*P*		0.514	0.474	0.001^*∗*^		0.458		0.559		

Group	Example number	Tumour diameter		Degree of differentiation		Pathological type			Growth	
		<5.0 cm	≥5.0 cm	High differentiation	Medium and low differentiation	Squamous cancer	Adenous squamous carcinoma	Papillary adenocarcinoma	The distal modular type	The proximal nodular type + diffuse type

There is extrawall vascular invasion	40	6 (15.00)	34 (85.00)	13 (32.50)	27 (67.50)	21 (52.50)	11 (27.50)	8 (20.00)	14 (35.00)	26 (65.00)
There is no extravascular invasion	91	61 (67.03)	30 (32.97)	34 (37.36)	57 (62.64)	44 (48.35)	30 (32.97)	17 (18.68)	59 (64.84)	32 (35.16)
*t/χ* ^2^		30.108		0.286		0.387			10.025	
*P*		0.001^*∗*^		0.593		0.824			0.002^*∗*^	

*Note.* TNM staging meets the criteria in the 8th edition TNM staging system for gastric cancer issued by UICC and AJCC. *P* < 0.05 indicates that the difference is statistically significant.

**Table 3:** Results of the logistic regression analysis.

Factors	*β*	SE	Walds	*P*	OR (95%CI)
T3∼T4	1.322	0.324	16.648	0.001^*∗*^	3.751 (1.988∼7.078)
Tumor diameter was ≥5.0 cm	1.065	0.305	12.193	0.001^*∗*^	2.901 (1.596∼5.274)
The proximal nodular type + diffuse type	1.214	0.411	8.725	0.001^*∗*^	3.367 (1.504∼7.535)

*P* < 0.05 indicates that the difference is statistically significant.

## Data Availability

The data used to support this study are available from the corresponding author upon request.
